# The Effects of Hedgehog Signaling Pathway on the Proliferation and Apoptosis of Melanoma Cells

**DOI:** 10.1155/2022/4984866

**Published:** 2022-01-04

**Authors:** Zhi-Peng Peng, Shan-Fu Huang, Jun-Jun Li, Xi-Ke Tang, Xi-Yue Wang, Hong-Mian Li

**Affiliations:** ^1^Dermatology Department, The Affiliated Nanning Infectious Disease Hospital of Guangxi Medical University and the Fourth People's Hospital of Nanning, Nanning 530023, China; ^2^Dermatology Department, The People's Hospital of Binyang County, Binyang 530405, China; ^3^Research Center of Medical Sciences, The People's Hospital of Guangxi Zhuang Autonomous Region & Guangxi Academy of Medical Sciences, Nanning 530021, China; ^4^Research Centre for Regenerative Medicine and Guangxi Key Laboratory of Regenerative Medicine, Guangxi Medical University, Nanning 530022, China

## Abstract

**Background:**

Studies have found that the abnormality of the Hedgehog signaling pathway is related to the occurrence and development of a variety of tumors, but the effect of this signaling pathway on melanoma cells is still unclear.

**Methods:**

This study aimed to discuss the effect of Hedgehog signaling pathway on the proliferation and apoptosis of human malignant melanoma A375 cells and explore its possible mechanism in the proliferation and apoptosis of melanoma cells. Different concentrations of Hedgehog signaling pathway inhibitor cyclopamine (5, 10, 20 and 40 *μ*M) were used to treat human melanoma A375 cells for 24, 48, and 72 h, and set a blank control group (0 *μ*M). Trypan blue cell counting method was used to detect cell viability. MTT method was used to detect the inhibition rate of cell proliferation. Transwell was used to detect cell invasion, and flow cytometry was used to detect cell apoptosis.

**Results:**

Through the trypan blue cell counting method and MTT experiment, it was found that the Hedgehog signaling pathway inhibitor cyclopamine has an inhibitory effect on the proliferation and viability of melanoma A375 cells (*P* < 0.05), and the proliferation inhibitory effect is enhanced with prolonged action time in a dose- and time-dependent manner. Transwell experiment showed that compared with the blank control group, the invasion and migration ability of the treated melanoma A375 cells are significantly reduced, and the difference is statistically significant (*P* < 0.05). Cell apoptosis experiment showed that compared with the blank control group, the apoptosis rate of A375 cells is significantly higher after treated by 40 *μ*M cyclopamine for 24 h, and the difference is statistically significant (*P* < 0.05). Gli1 and Bcl-2 protein are highly expressed in melanoma A375 cells, and their expressions show a downward trend (*P* < 0.05) after being treated by cyclopamine.

**Conclusion:**

Cyclopamine inhibits cell proliferation and induces cell apoptosis by downregulating Gli1. Hedgehog signaling pathway can be used as a new target for the treatment of malignant melanoma, and multiple measures can be used to inhibit the signaling pathway to achieve a therapeutic effect.

## 1. Introduction

Melanoma is one of the most aggressive cancers, and its incidence has been increasing globally in the past two to three decades [1, 2]. These tumors originate from the melanocyte lineage and cannot be cured after metastasis. With the development of science and technology, although researchers have made progresses and breakthroughs in the treatment of melanoma, the overall median survival time of melanoma patients is only 4–6 months [2–4]. Therefore, it is of great significance for the clinical treatment of melanoma cells to fully understand the occurrence and development mechanism of melanoma cells at the genetic level, discover its downstream target genes, and then find some new effective drugs to inhibit the proliferation and metastasis of melanoma cells.

In the early stage of the experiment, we analyzed the differentially expressed genes of melanoma (melanoma) by using human genome-wide microarray and screened 346 signaling pathways closely related to tumorigenesis, among which the Hedgehog signaling pathway in melanoma A375 cells was in a highly activated state, indicating the abnormal activation of this signaling pathway was closely related to the occurrence of melanoma.

The evolutionarily conserved Hedgehog (Hh) signaling pathway was first discovered by Christiane Nüsslein-Volhard and Eric Wieschaus [5] in *Drosophila melanogaster*, and it was found to play a key role in embryonic development. Hedgehog signaling pathway has two different signal activation pathways, which are called classical pathway and nonclassical pathway, respectively [6]. In the classical pathway, the SHH ligand recognizes and binds to the Ptch receptor and then prompts the release of the Smo protein, triggering an intracellular cascade reaction. The final result is activating the transcription factors of the Gli family, shifting its nuclear localization, affecting the expression of downstream genes, and thus regulating the biological functions of cells [7, 8]. In the nonclassical pathway, the Hedgehog signaling pathway is activated in an independent ligand-receptor binding mode, such as mutations in common pathway genes, and changes in the activity or function of Gli family transcription factors [9, 10]. The HH pathway remains dormant in adult tissues, but it is activated when needed, such as in tissue repair and regeneration [11]. However, its abnormal activation is related to cancer development and progression, tumor recurrence, and drug resistance treatment. Therefore, understanding the paradigm of HH signaling is essential for designing new tools for the treatment of cancers associated with abnormal HH signaling.

Based on the above analysis, this study mainly used cyclopamine, a specific blocker of the downstream molecule SMO of the Hedgehog signaling pathway, to treat cells, inhibit the activity of the signaling pathway, and observe its effects on the proliferation and apoptosis of melanoma A375 cells, to further clarify whether the Hedgehog signaling pathway is involved in the occurrence and development of melanoma A375 cells and provide certain theoretical support for the future clinical treatment of melanoma.

## 2. Materials and Methods

### 2.1. Materials

#### 2.1.1. Cells

The human melanoma cell line A375 used in this study was purchased from the Chinese Academy of Sciences (Shanghai). The A375 cells needed to be cultured in a 5% CO2 humidified incubator with RPMI-1640 medium supplemented with 10% heat-inactivated bacteria. The incubator was kept at 37°C.

#### 2.1.2. Reagent

Fetal bovine serum and RPMI-1640 medium were purchased from GIBCO, USA; trypsin-EDTA digestion solution, MTT, and DMSO were purchased from Sigma, USA; penicillin streptomycin mixture and OPTI-MEM were purchased from Solarbio, USA; Tris balanced phenol was purchased from Thermos, USA; 60 mm/100 mm Petri dishes and 6/12/24/48/96-well cell culture plates were purchased from CORNING, USA; RIPA lysate and BCA protein concentration kits were purchased from Beyotime; antibodies and protease inhibitors were purchased from Proteintech.

### 2.2. Methods

#### 2.2.1. Cell Culture

In this study, all the cell lines were cultured in RPMI-1640 medium (BI, USA) containing 10% fetal bovine serum and 1% penicillin/streptomycin double antibody after resuscitation. The cells were cultured in an incubator, and the culture conditions were 37°C and 5% CO_2_.

#### 2.2.2. Trypan Blue Cell Counting Method

1. When the cells were cultured to the logarithmic growth phase, they were redigested, put into a 6-well plate with a cell density of 1 × 10^4^/cm^2^ per well, and then placed in a 37°C cell incubator to continue culturing
2. When the cell density reached 70%–80%, cyclopamine of different concentration gradients (5, 10, 20, 40 *μ*M) was added into the 6-well plate and placed in a 37°C incubator for 24 h
3. After 24 h, the cells were digested, centrifuged, resuspended to yield cell suspension, and mixed with 0.4% trypan blue solution at a ratio of 9 : 1 (the final concentration was 0.04%)
4. The cells were counted under a microscope according to the cell counting principle, the number of dead cells and living cells, respectively, was recorded, and then the living cell rate was calculated according to living cell rate (%) = total number of living cells/(total number of living cells + total number of dead cells) × 100%

#### 2.2.3. MTT Experiment

1. The cells were cultured and the cell state was observed under a microscope. When the cell density reached 80%–90% and the cells were in good state, the cells with 0.25% trypsin were digested until the cells came off from the Petri dish. 1 mL of cell culture medium was used to terminate the digestion reaction, and the culture medium was resuspended. A pipette was used to suck 10 *μ*L of cell culture medium and the cells were counted. The cells were serially diluted and then evenly put it into a 96-well cell culture plate, with 1,000 cells in each well and placed in a 37°C cell incubator to continue culturing.
2. After the cells were placed into 96 wells, 100 *μ*L of cyclopamine medium was added with different concentrations to each well (the concentration gradients of the experimental group were 5, 10, 20, and 40 *μ*M, respectively, and the control group was added with normal medium). We set 5 replicate wells for each concentration, and the control group was the same as above. Then, we placed it in a 37°C cell incubator to continue culturing.
3. After 24 h, the drug effect under a microscope was observed, and then 20 *μ*L of MTT solution (with the concentration of 5 mg/mL) was added to each well. After culturing for 4 h, the 96-well cell culture plate containing the MTT solution was taken out. A pipette was used to discard the culture medium in each well, and then 150 *μ*L of DMSO was added to each well and kept for 10 min at room temperature. We put the 96-well cell culture plate into a microplate reader and measured the absorbance of the solution at 490 nm wavelength and saved the experimental data at that point in time.
4. We took the experimental time on the first day as the initial time point and then performed the above operations repeatedly on the cell culture plate after 24 h, 48 h, and 72 h, respectively, to obtain the 5-day experimental data. We sorted the 5-day experimental data, used GraphPad Prism 8 software to process the data, and gained the cell proliferation curve by analyzing the data.

#### 2.2.4. Cell Apoptosis Experiment

1. The cells that were in good state were taken and had just adhered to the wall, and 40 *μ*M cyclopamine medium was added and cultured for 24 h, 48 h, and 72 h, respectively. Then the cells were treated uniformly in the following manner.
2. They were rinsed gently with 1 × PBS working solution for 2–3 times; then 0.25% EDTA-free trypsinized cells to the cell Petri dish to digest the cells were added. After the cells were digested completely, the cell culture solution containing 10% FBS was added to terminate the digestion reaction. The cell suspension was transferred to a 1.5 mL sterile Ep tube and placed it on ice.
3. We put the Ep tube containing cell suspension in a centrifuge, set the centrifuge to 1000 rpm/min, and centrifuge at room temperature for 10 min. We discarded the supernatant after the centrifugation was complete.
4. 500 *μ*L of precooled 1 × binding buffer was added to the Ep tube to resuspend the cells and centrifuged again at 1000 rpm/min for 5 min at room temperature, and the supernatant was discarded after centrifugation.
5. A pipette was used to add 100 *μ*L of 1 × binding buffer, respectively, to resuspend the cells. The cells in the control group were divided into three subgroups, namely, the blank group without treatment, the PI single-stained group, and Annexin V single-stained group. The cells in the experimental group were dual-stained with PI and Annexin V. 2.5 *μ*L of each staining solution dropwise was added and stained at room temperature for 15 min away from light, with Annexin V staining for 10 min and PI staining for 5 min.
6. Then, 400 *μ*L of 1 × binding buffer was added to each Ep tube, the cell suspension was transferred to the sample tube dedicated for flow cytometry, computer testing was performed on the flow cytometer, the results were analyzed, and the analyzed results were input into the GraphPad Prism 8 software. After data processing, a histogram of cell apoptosis was obtained.

#### 2.2.5. Transwell Experiment

1. The Transwell experiment was carried out in a 24-well plate. The cells in the logarithmic growth phase were taken. The cells for counting were digested, centrifuged, and resuspended. The cells with 10% FBS-free cell culture medium and 40 *μ*M serum-free medium to the appropriate concentration were diluted, generally 2.5 × 10^5^ cells/mL.
2. 200 *μ*L of the diluted cell suspension (without serum) was taken and added to each cell compartment to gain a cell density of 5 × 10^4^ cells/mL. The experimental group and the control group each repeated three groups. 700 *μ*L of cell culture medium containing 15% FBS in the lower layer of each cell compartment was added. Be careful to operate gently to prevent air bubbles from forming in the lower layer of the cell compartments.
3. Then, we placed the cell compartments in a 37°C, 5% CO2 cell incubator for culture. After culturing for 24 h, we took out the cell compartments for the cell migration experiment. Since the cell perforation time was longer in the cell invasion experiment, we took it out after culturing for 48 h. We took out the cell compartments at the specified time, wiped off the excess cells with a cotton swab, washed them with 1 × PBS, fixed them for 30 min with 4% paraformaldehyde, stained them with crystal violet for 30 min, rinsed them gently with running water, observed and took pictures under a microscope, counted the number of migrated cells, and saved the data.
4. In the cell invasion experiment, we fully mixed 100 *μ*L of Matrigel gel with 500 *μ*L of serum-free medium, drew 50 *μ*L into the cell compartments, and cultured it in an incubator for 4 h. The remaining steps were the same as above.

#### 2.2.6. Western Blotting Experiment

1. The experimental cells were spread evenly into a 6-well plate, cultured overnight, and then treated with drugs. After 48 h, we washed it with 1 × PBS for 2–3 times. We scraped off the cells with a cell brush and placed them in a 1.5 mL centrifuge tube. We put the tube on ice. After centrifugation, we discarded the supernatant, added RIPA lysate to the pellet, sonicated the cells, and repeated 2–3 times to ensure the protein can be fully lysed. After the sonication, we centrifuged the cells for 15 min and aspirated the supernatant to obtain protein sample.
2. We used the BCA kit purchased from Beyotime to measure the concentration of the obtained protein. According to the sample size, we took the corresponding sample volume and an equal volume of 1 × loading and boiled it in boiling water for 5 min to denature the protein.
3. We added the sample to the preprepared 12.5% SDS-PAGE gel well, put on the electrophoresis cover, set the electrophoresis instrument to 80 V for 30 min, and switched to 100 V for 1 h after the protein sample band entered the separation gel. After the target band completely ran away, we cut the gel and transferred it to the membrane according to the operation instructions.
4. The transfer needed to be carried out in an ice bath at a constant current of 220 mA for 60 min. After the transfer was completed, we put the membrane in the preprepared 5% milk medium and sealed for 1 h. After that, we put the membrane into the 1 × TBST washing solution and rinsed 3 times, 10 min each time. We checked the antibody instructions, diluted the antibody proportionally with TBS buffer, placed the membrane in the diluted antibody solution, and incubated overnight in a refrigerator at 4°C.
5. We washed the membrane 3 times with 1 × TBST washing solution on the next day, 10 min each time. We transferred the membrane to the secondary antibody (horseradish peroxidase-labeled goat anti-rabbit IgG, 1 : 5000, Beijing CWBIO) and incubated on a shaker for 1–2 h. After the secondary antibody incubation, we washed it with 1 × TBST washing solution 3 times, 10 min each time. Finally, we dropped appropriate volume of ECL luminescent liquid evenly on the PVDF membrane according to the size of the membrane, exposed by a gel imager, and collected images through the Image studio software. We adjusted the strength of the target protein band after exposure, marked the experiment date, name, and protein sample loading sequence, and saved the images.

### 2.3. Statistical Processing

The statistical software SPSS21.0 was used to analyze the data. The measurement data were expressed as mean ± standard deviation (mean ± SD). The independent sample *t*-test was used for the comparison between two groups, and the one-way analysis of variance was used for the comparison between multiple groups. *P* < 0.05, and the difference was statistically significant.

## 3. Results

### 3.1. The Effect of Cyclopamine on Cell Proliferation and Viability

After the cells were treated with cyclopamine, it can be observed under microscope that the cell growth was significantly slowed down and the cells became smaller; some had shrunk cell membranes, nuclear pyknosis, reduced or disappeared intercellular junctions, and more suspended single cells. The higher the concentration and the longer the action time, the more prominent these changes. Through the trypan blue cell counting method, it was found, as shown in Figure 1(a), the cyclopamine at a concentration of 5–40 *μ*M has a significant inhibitory effect on cell proliferation and a certain concentration dependence was shown. Compared with the control group, the difference is statistically significant (*P* < 0.05). Cyclopamine of different concentrations were used for MTT experiment and cultured for 24 h, 48 h, and 72 h, respectively. It was found that, as shown in Figure 1(b), the cell proliferation and viability decrease significantly, and the difference is statistically significant compared with the control group (*P* < 0.05  ). This showed that with the increase of the concentration of cyclopamine (within a certain range) and the increase of the reaction time, the cell viability gradually decreases. Among all the concentrations, the effect of 40 *μ*M cyclopamine is most obvious (*P* < 0.01), so the following experiments were carried out at this concentration.

### 3.2. The Effect of Cyclopamine on Cell Apoptosis

In order to analyze whether the Hedgehog signaling pathway affects the apoptosis of melanoma cells, the apoptosis experiment was carried out on the cells of the experimental group and the control group by dual staining.  Figure 2(a) shows the apoptosis of the cells in the control group and the experimental group. According to the figure, different quadrants represent different meanings. The cells in the upper left quadrant are the percentage of dead cells to the total number of cells, and the cells in the lower left quadrant are the percentage of viable nonapoptotic cells to the total number of cells. The cells in the upper right quadrant are the percentage of nonviable apoptotic cells to the total number of cells, and the cells in the lower right quadrant are the percentage of viable apoptotic cells to the total number of cells. The percentages of cells in the upper right and lower right quadrants to the total number of cells are added to get the sum percentage of apoptotic cells. It can be seen from the figure that the percentage of nonviable apoptotic cells in the experimental group with the addition of cyclopamine is significantly higher than that in the control group. Subsequently, the experimental data was sorted and input into the GraphPad Prism8 software, and Figure 2(b) was obtained through analysis, which shows the percentage of apoptotic cells of the experimental group and the control group. According to the experimental results, it can be seen that compared with the control group, the nonviable apoptosis rate of the experimental group is upregulated, with no significant change in the viable apoptosis rate. In addition, the percentage of apoptotic cells in the experimental group are upregulated, and the difference is statistically significant (*P* < 0.05). After collating the experimental results, it can be concluded that after the signaling pathway is blocked, the apoptosis rate of melanoma cells increases.

### 3.3. The Effect of Cyclopamine on Cell Invasion and Migration

Next, the study verified the effect of the Hedgehog signaling pathway on the invasion and migration of A375 cells through cyclopamine. According to Figures 3(a) and 3(b), it can be seen that the cells treated with cyclopamine have fewer migrating and invading cells than NC group, and the difference between the two groups is statistically significant (*P* < 0.05). These results indicate that cyclopamine can effectively inhibit the migration and invasion of A375 melanoma cells by blocking the HH signaling pathway in A375 melanoma cells.

### 3.4. The Effect of Cyclopamine on the Expression of Gli1 and Bci-2 Protein in A375 Cells

As shown in Figures 4(a) and 4(b), the results of western blotting showed that the protein expression levels of Gli and Bcl-2 in melanoma A375 cells are not low, but after treatment with cyclopamine (at a concentration of 40 *μ*M), the protein expression levels of Gli and Bcl-2 present a downward trend (*P* < 0.05). At the same time, in Figure 4(b), the left images show the typical and atypical activation pathways of the HH signaling pathway in melanoma: SOX2 and BRD4 form a complex, and BRD4, by interacting with acetylated histones in the proximal region of the *GLI1* promoter, induces RNA polymerase 2 activity and transcriptional activation of *GLI1*. In the right images, the SMO antagonist cyclopamine inhibits canonical HH signaling, whereas it induces BRD4 degradation with consequent inhibition of *GLI1* transcription.

## 4. Discussion

Studies have shown that skin melanoma is based on the malignant transformation of melanocytes and is the most aggressive skin cancer, with a poor prognosis in the advanced stage [12, 13]. In recent years, the incidence of melanoma has gradually increased, so it has become an urgent clinical problem to develop early diagnosis means and treatment methods for melanoma as soon as possible. Many signaling pathways have been found to be involved in the occurrence and development of tumors, such as Wnt/*β*-catenin, Notch, and HH signaling pathway [14]. The high-throughput data in the early stage of the laboratory have showed that the abnormal activation of the HH signaling pathway is closely related to the occurrence of melanoma. Blocking the pathway may be a treatment method for melanoma. Therefore, this study mainly explores the effect of Hedgehog (HH) signaling pathway on the proliferation and apoptosis of melanocytes [15].

A large number of previous studies have proved that the Hedgehog (HH) signaling pathway is closely related to human cancer [16]. For example, the key role of HH signaling in the development of basal cell carcinoma (BCC) has been convincingly proven in gene mutation analysis, mouse models, and BCC clinical trials using HH signaling inhibitors [17]. However, due to the lack of genetic changes in HH pathway genes [18] and the lack of mouse models of HH signal-mediated melanoma [19], the activity of HH pathway in the occurrence of melanoma has not been discovered until recent years [20]. The HH signaling pathway is a conservative pathway that directs the mode of embryogenesis through temporal and spatial regulation of cell proliferation and differentiation [8]. During development, once the HH signal is lost, some physiological processes in human and mice may become severely abnormal [21]. In adults, HH signals mainly exist in stem cells, which are mainly responsible for regulating the homeostasis, repair, and regeneration of tissues [9]. In this study, we mainly explored the effect of the Hedgehog signaling pathway on the proliferation and apoptosis of melanoma cells. Previous studies have also proved that cyclopamine is an effective drug for HH signaling, and it has no side effect on other parts of the body [22–24]. Based on this, the main experimental method is to use cyclopamine, a specific blocker of the downstream molecule SMO of the Hedgehog signaling pathway, to treat cells, inhibit the activity of the signaling pathway, and observe its effects on the proliferation and apoptosis of melanoma A375 cells, to further clarify whether the Hedgehog signaling pathway regulates the proliferation and apoptosis of melanoma A375 cells.

In this study, we found that the growth of melanoma A375 cells significantly slow down, the cells become smaller and rounder, and the surface membrane shrinks after treatment with cyclopamine. At the same time, the higher the concentration and the longer the action time and the more prominent these changes. The results of the trypan blue cell counting method and the MTT experiment showed that the melanoma A375 cells treated with the HH signaling pathway blocker cyclopamine have a decreased proliferation ability compared with the control group. The apoptosis experiment of flow cytometry showed that the apoptosis rate is increased. Based on the above results, it can be concluded that the HH signaling component supports the proliferation of melanoma A375 cells and that blocking the signaling pathway can inhibit the proliferation and growth of the cells and promote apoptosis. This is similar to conclusions drawn in tumors of pancreatic cancer, gastric cancer cell lines, and so on. At the same time, according to the results of Western blotting, the expression of Gli1, a key factor in the downstream of SMO in the HH signaling pathway, and the expression of apoptosis-related protein Bcl-2 decrease, indicating that these effects of A375 cells may be regulated by the HH signaling pathway.

## 5. Conclusions

In summary, the abnormal activation of the HH signaling pathway is closely related to the occurrence, development, metastasis, and prognosis of tumors. It is abnormally activated in melanoma A375 cells. By specifically blocking this signaling pathway, it is found that cell proliferation, invasion, and migration are inhibited, and the apoptosis rate is increased. Therefore, blocking the HH signaling pathway may be able to achieve targeted treatment of melanoma. Of course, more work is needed to confirm how this signaling pathway regulates melanoma and provide more detailed theoretical support for the clinic.

To sum up, we used HH signaling pathway inhibitor cyclopamine to treat melanoma cells and found that by specifically blocking the HH signaling pathway, the proliferation, invasion and migration of melanoma A375 cells are inhibited, and the rate of apoptosis is increased. Therefore, this study provides a method that may be able to achieve targeted treatment of melanoma by blocking the HH signaling pathway. Of course, more work is needed to confirm how this signaling pathway regulates melanoma and provide more detailed theoretical support for clinical treatment.

## Figures and Tables

**Figure 1:** The effect of different concentrations of cyclopamine on the proliferation and viability of A375 cells at different times. Note: mean ± SD (*n* = 5). *P* < 0.05 versus control group.

**Figure 2:** The effect of 40 *μ*M cyclopamine on A375 cell apoptosis. Note: mean ± SD (*n* = 3). *P* < 0.01 versus 0 h group. *P* < 0.05 versus 24 h/48 h group.

**Figure 3:** The effect of 40 *μ*M cyclopamine on the invasion and migration ability of A375 cells. Note: random visual view under 200 times microscope; mean ± SD (*n* = 3). *P* < 0.05 versus control.

**Figure 4:** (a) The effect of 40 *μ*M cyclopamine on the expression of Gli1 protein and Bcl-2 protein in A375 cells; (b) schematic representation of canonical and noncanonical HH signaling and their inhibition by cyclopamine. *Note.* Mean ± SD (*n* = 3). *P* < 0.05 versus control group.

## Data Availability

The analyzed data sets generated during the study are available from the corresponding author upon reasonable request.
